# Lineage Contribution of PDGFR*α*-Expressing Cells in the Developing Mouse Eye

**DOI:** 10.1155/2021/4982227

**Published:** 2021-07-02

**Authors:** Deyi Zhuo, Yumei Diao, Xiaoqi Li, Yifei Huang, Liqiang Wang

**Affiliations:** Department of Ophthalmology, The Third Medical Center of Chinese PLA General Hospital, Beijing 100853, China

## Abstract

PDGFR*α* signaling is critically important in ocular development. Previous data on PDGFR*α* lacks an expression map with high spatial and temporal resolution and lineage information. In this study, we aim to present a detailed PDGFR*α* expression and lineage map from early embryogenesis to adulthood. PDGFR*α*-CreER; mT/mG reporter mice were analyzed. mEGFP-positive cells contributed to multiple ocular lineages in a spatiotemporally regulated manner. A dynamic PDGFR*α* expression was identified in corneal stromal cells, lens epithelial cells, lens fiber cells, and retinal astrocytes during the entire period of eye development, while PDGFR*α* expression in retinal astrocytes from E17.5 onwards and in Müller glial cells was identified within two weeks after birth. By revealing detailed characterization of gene expression and function, we present a comprehensive map of PDGFR*α*-expressing cells in the eye for a better understanding of PDGFR*α* signaling's role during eye development.

## 1. Introduction

The vertebrate eye is a very complex organ, and its development has been widely characterized [1, 2]. Ocular development commences during gastrulation with the single central eye field (late gastrula stage). The singular eye field subsequently splits into two lateral parts to form the optic vesicle and the lens placode (placode stage, E9.5 in the mouse) [3]. Shortly afterwards, the lens placode invaginates to a lens pit, which occurs coordinately with optic cup invagination (lens pit stage, E10.5 in the mouse) [4]. At E11.5 in the mouse (optic cup stage), the future cornea, lens, and retina become visible. The anterior eye tissues evolve to form the surface ectoderm, lens, and corneal epithelium, while the surrounding neural crest cells give rise to the corneal stroma and corneal endothelium [5]. The retina comes from the underlying neural ectoderm. Development of the eye depends on the proper function of various transcription factors and signaling pathways [6, 7].

The PDGF family consists of two receptor genes, PDGFR*α* and PDGFR*β*, and four ligand genes, PDGF-A, PDGF-B, PDGF-C, and PDGF-D [8–10]. PDGF-A and PDGF-C exclusively bind and activate PDGFR*α* in vivo [11, 12]. PDGFR*α* signaling has a broader role in embryogenesis and function during organogenesis, such as lung alveogenesis, intestinal villus morphogenesis, hair morphogenesis, testis spermatogenesis, and oligodendrogenesis [13]. PDGFR*α* signaling is also essential in ocular development, particularly involving the cornea, lens, and retina. PDGFR*α* null embryos display developmental abnormalities in multiple organs and systems, and this could even result in embryonic lethality [14–16]. Homozygous Patch mutation in mice, which is a deletion of the gene encoding PDGFR*α*, presents a thinned cornea and a decreased number of fiber cells within the mutant lens [17]. A detailed analysis of the PDGFR*α* null lens shows retarded elongation of primary lens fiber cells, anteriorly shifted transitional zone, and smaller lens size [18]. Overexpression of PDGF-A under the *α*A-crystallin promoter results in lenticular defects and hyperplasia of retinal astrocytes [19, 20].

PDGFR*α* expression has been detected in the embryonic eye using immunohistochemistry (IHC) and/or RNA in situ hybridization (ISH) in early studies [19]. However, ISH is technically difficult to perform on adult tissues [21]. Moreover, IHC-based expression studies often cannot explain the potential fate and lineage of the cells that express the gene of interest [22]. In addition, only very few studies have focused on PDGFR*α*'s role in the embryonic and postnatal eye simultaneously. Due to limited spatial and temporal resolution, the existing data is not able to provide sufficient information as to which ocular lineage(s) expresses PDGFR*α* or its expression duration in that lineage. Therefore, the spatiotemporal requirement for PDGFR*α* in ocular development remains to be elucidated.

In this study, we map the detailed expression and lineage analyses of PDGFR*α* from embryonic to adult ages in the eye, aiming at comprehensively understanding PDGFR*α* signaling during eye development.

## 2. Materials and Methods

### 2.1. Animals

PDGFR*α*-CreER^T2^ transgenic mice are crossmated with ACTB-tdTomato, -EGFP reporter mice in order to generate PDGFR*α*-CreERT2; mT/mG mice [23]. Genotyping is performed as previously described. To genotype the CreER^T2^ allele, PCR Genotyping is performed with genomic DNA extracted from tail tip with sense primer (5′-ATCCCATCAGCTCACAGACTTCGGA-3′) and antisense primer (5′-GCTCTTCGCCCTTAGACACCATAGG-3′) specific for the CreER^T2^. To detect the wild-type PDGFR*α* allele, sense primer (5′-ATCCCATCAGCTCACAGACTTCGGA-3′) and antisense primer (5′-CAAGAGGCAACACGGATAAAGTTCA-3′) are used for PCR. The PCR products for CreER^T2^ wild-type and knock-in alleles are 353 bp and 243 bp, respectively. To genotype mice expressing the mT/mG transgene, three primers are used: mT/mG wild type 5′-CTCTGCTGCCTCCTGGCTTCT-3′, mT/mG wild type 5′-CGAGGCGGATCACAAGCAATA-3′, and mT/mG 5′-TCAATGGGCGGGGGTCGTT-3′. The PCR products for mT/mG wild-type and knock-in alleles are 330 bp and 250 bp, respectively. All procedures regarding the use and the handling of animals were approved by the Institutional Animal Care and Use Committee of the General Hospital of Chinese PLA. The approval number from Animal Experiment Committee is SQ2020112.

### 2.2. Tamoxifen Administration

The day of vaginal plug formation is designated as E0.5. Pregnant females receive a single intraperitoneal injection with tamoxifen (Sigma) at 50 *μ*g/g body weight (20 mg/mL in 90% corn oil/10% 4-OHT). Pregnant female mice are treated with tamoxifen at E9.5, E11.5, E13.5, E15.5, and E17.5 of gestation according to the needs. Tamoxifen's postnatal intraperitoneal dosage is 180 *μ*g/g/day for 3 days. For lineage tracing experiments, 6~8 embryos are used at each time point.

### 2.3. Immunofluorescence

Cryosections of the eyeball (8-10 *μ*m) are incubated at room temperature in blocking solution (10% normal goat serum+0.3% Triton X-100 in PBS) for 45 minutes. Antibodies used for immunofluorescence are as follows: rabbit anti-ALDH3A1 (1 : 100; Proteintech), mouse anti-*α* B crystallin (1 : 200; Abcam), rabbit anti-GFAP (1 : 500; Abcam), rabbit anti-BRN3A (1 : 100; Abcam), rabbit anti-Sox9 (1 : 100; Abcam), rabbit anti-glutamine synthetase (1 : 400; Abcam), and rabbit anti- PDGFR*α* (1 : 500; Abcam). Secondary antibodies used are donkey-anti-rabbit Alexa Fluor-647 (1 : 400, Abcam) and goat-anti-mouse Alexa Fluor-647 (1 : 400, Abcam). All-section immunofluorescence data shown are imaged and photographed on a Zeiss spinning-disk confocal microscope (SDCM).

### 2.4. RNA Isolation and Quantitative PCR (qPCR)

Total RNA is isolated with a RNeasy Micro kit (Qiagen) and reverse transcribed using a First-Strand cDNA Synthesis kit (Servicebio) according to the manufacturer's protocol. qPCR is performed using 400 ng of cDNA, 2× SYBR Green qPCR Master Mix (Servicebio), and the following primers: PDGFR*α*, forward primer CCTCATCTCCTGCCAGCTCTT, and reverse primer CTCCTCACTTCTGATTTCCACG.

### 2.5. Statistical Analysis

Data is presented as mean ± SEM. Differences between calculated averages are considered significant when *P* < 0.05 by Student's *t*-test. qPCR results between the different time points are studied by using a two-way ANOVA with Tukey's multiple comparisons test.

## 3. Results

### 3.1. PDGFR*α*-Expressing Cells in the Adult Mouse

When we perform tamoxifen administration on adult mice and collect eyeballs 7 days later, we observe the expression of PDGFR*α* in their adipose cells (Figures 1(a) and 1(e)), bone marrow stromal cells (Figures 1(b) and 1(f)), kidney mesangial cells (Figures 1(c) and 1(g)), and hepatic stellate cells (Figures 1(d) and 1(h)). In the eye of an adult mouse, mEGFP-positive cells are observed in the cornea, lens, iris, ciliary body, drainage structures, retina, optic nerve, and sclera (Figure 1(i)). mEGFP-positive cells in the iris, ciliary body, drainage structures, and sclera are most likely to be stromal cells. The expression map of PDGFR*α* cells and their descendants in the cornea (Figure 1(j)), lens (Figure 1(k)), and retina (Figure 1(l)) are investigated in more detail. mEGFP-positive cells are located mainly in the corneal stroma, lens epithelial and differentiating fibers, and the retina's ganglion cell layer (GCL). Several antibodies, including ALDH3A1 (a corneal crystallin), *α*B crystallin (a lens crystallin), and GFAP (a known glial marker), are used to identify mEGFP-positive cells in the eye. Staining of eye sections demonstrates that corneal stromal cells, lens epithelial, fiber cells, and retinal astrocytes contained mEGFP.

### 3.2. PDGFR*α*-Expressing Cells Contribute to Corneal Lineages in the Embryonic and Postnatal Stages

After a single dose of tamoxifen administration at E11.5, embryos that are harvested at E12.5 show the mEGFP-labeled cells are weakly dispersed in the prospective cornea, originating from the periocular mesenchyme (POM) (Figure 2(a)). When the eyes are harvested at P0 (Figure 2(i)) after a single dose of tamoxifen at E11.5, mEGFP-positive cells are shown to be confined to the corneal stroma. Other POM-contributing structures including the sclera, iris, and ciliary body, meanwhile, are found to contain mEGFP-positive cells. When these E11.5 tamoxifen-induced embryos are harvested at P14 (Figure 3(a)), it is confirmed that mEGFP-positive cells in the cornea are keratocytes (Figure 3(b)). A similar expression pattern is seen with embryos induced with a single dose of tamoxifen at E13.5~E14.5 (Figures 2(b), 2(j), and 3(f)), when the POM cells between the anterior epithelium of the lens vesicle and the surface epithelium condense to form several flat layers that are separated from each other by a loose fibrillar extracellular matrix. In the stage when the posterior POM cells closest to the lens are flattened to form an endothelial monolayer (E15.5~E16.5), PDGFR*α* expression in the corneal stroma is induced to higher levels compared to previous time points by a single dose of tamoxifen. (Figures 2(c), 2(k), and 3(j)). When the eyes are administrated with tamoxifen at E17.5 (Figures 2(d), 2(l), and 3(n)), mEGFP-positive cells in the cornea are further increased and restricted to the corneal stroma.

For the analysis of the postnatal stages of eye development, four time points (P1, P3, P7, and P14) are selected to inject tamoxifen, and mouse eyes are harvested at P30. After birth, the PDGFR*α* expression is similar to E18.5 (Figures 4(b), 4(f), and 4(j)). As the eyelids start opening between P12 and P14 (Figure 4(n)), the corneal stroma significantly thickens, and the keratinocytes' nuclei continues to flatten with chromatin condensation. The flattened and matured keratinocytes stay mEGFP positive. At the latest analyzed time point (P60), cornea development is completed. At this stage, PDGFR*α* is still expressing in corneal stromal cells (Figure 1(j)).

Our results, therefore, indicate that although there are some differences in expression levels, PDGFR*α* expression is persistent not only in early corneal mesenchymal progenitors at embryonic stages but also in the differentiated keratocytes in adulthood.

### 3.3. PDGFR*α*-Expressing Cells Contribute to Lens Lineages in the Embryonic and Postnatal Stages

At E12.5 (Figure 2(a)), when the lens vesicle is filled by the primary lens fibers, the epithelial cells divide and move to the lens equator (LE), mEGFP-positive cells are induced in the germinative zone, and lens bow (equator) after a single dose of tamoxifen at E11.5. Eyes harvested at P0 (Figure 2(i)) or P14 (Figure 3(c)) after a single dose of tamoxifen at E11.5 show PDGFR*α* expression in the lens epithelial cells and lens primary and secondary fiber cells. At E14.5, when the primary lens fibers elongate to close the lumen of lens vesicle, the PDGFR*α* expression is induced to be found in the lens epithelial cells after a single dose of tamoxifen at E13.5 (Figure 2(b)). We also detect PDGFR*α* expression in the majority of lens epithelial cells and their newly differentiated secondary lens fiber cells after a single dose of tamoxifen at E13.5, followed by consecutive days without treatment until P0 (Figure 2(j)) or P14 (Figure 3(g)). After a single dose of tamoxifen administration at E15.5, when the epithelial cells differentiate into secondary lens fiber cells, PDGFR*α* expression is induced in the lens epithelial and secondary fiber cells both in the short-term tracing experiments and long-term tracing experiments (Figures 2(c), 2(k), and 3(k)). The PDGFR*α* expression pattern of embryos induced at E17.5 and harvested E18.5 or later (Figures 2(d), 2(l), and 3(n)) is similar to those of embryos induced at E15.5.

As a result, mice induced at the postnatal stage (P1, P3, P7, and P14) and harvested at P30 exhibit mEGFP labeling of the entire lens epithelial cells and their differentiated lens secondary fiber cells (Figure 3), similar to E17.5-tamoxifen-induced embryos (Figures 4(c), 4(g), and 4(k)). Interestingly, at P14 (Figure 4(o)), when the centre of the lens is free of cellular organelles, such as nuclei and mitochondria, fewer mEGFP-positive cells are in the secondary lens fibers and anterior lens epithelium than P1~P7. In adult eyes (P60) after tamoxifen administration for 3 consecutive days, the expression of PDGFR*α* is confined to the lens epithelial cells, most of which is located in the lens bow (Figure 1(k)).

Collectively, PDGFR*α* expression in the lens lineages is constant and presents all throughout the ages examined, whereas its expression levels in the lens epithelial cells and fiber cells decrease markedly in adults.

### 3.4. PDGFR*α*-Expressing Cells Contribute to Retinal Lineages in the Embryonic and Postnatal Stages

At E11.5, when the retina's two layers (outer and inner layers) are closely attached, we administer a single dose of tamoxifen. One day later, embryos are harvested, and the results show that mEGFP-positive cells are not detected in the retina (Figure 2(a)), even after birth (P0 and P14 collecting eyes). Embryos induced at E13.5 and harvested at E14.5 show that PDGFR*α* is not expressed in the retina (Figure 2(b)), and we fail to detect any mEGFP-positive cells in the neuroblastic layer (NBL), ganglionic cell layer (GCL), or inner plexiform layer (IPL) in E13.5 tamoxifen-induced embryos harvested at P0 (Figure 2(j)). However, the retinas harvested at P14 (Figure 3(h)) show dispersed PDGFR*α* expression in the nerve fiber layer (NFL), and these mEGFP-positive cells are colabeled with GFAP (astrocytes). The PDGFR*α* expression pattern of E15.5 tamoxifen-induced embryos (Figures 2(c), 2(k), and 3(l)) is similar to E13.5 tamoxifen-induced embryos. The mEGFP-positive cells in the retina are first detected at E18.5 harvested embryos after a single dose of tamoxifen at E17.5 (Figure 2(d)). When the eyes are harvested at P0 (Figure 2(l)) after a single dose of tamoxifen at E17.5, it shows that PDGFR*α* expression is confined to the centre of the retinal nerve's fiber layer. However, mEGFP-positive cells migrate to the retina's periphery at P14 harvested eyes (Figure 3(p)). Moreover, mEGFP-positive cells will not reach the periphery of the retina until P7 (data not shown).

In the postnatal retina, a completely different PDGFR*α* expression pattern is observed. In neonatal mice tamoxifen induced at P1, P3, and P7 and harvested at P30 (Figures 4(d), 4(h), and 4(l)), retinal astrocytes stay mEGFP positive in the nerve fiber layer, and some cells with radial fiber morphology also express mEGFP. Müller glial cells labeled by Sox9 and glutamine synthetase coexpress mEGFP. However, their expression decreases, and when embryos induced at P14 and harvested at P30 (Figure 4(p)), such expression is only visible in the nerve fiber layer, whereas they have vanished in the Müller glial cells. After tamoxifen administration for 3 consecutive days in adults (Figure 1(l)), PDGFR*α* expression is only present in retinal astrocytes.

Overall, our analyses suggest that PDGFR*α* is expressed in the astrocyte precursor cells that give rise to retinal astrocytes from E17.5 to adult stages, and a small portion of immature Müller glial cells within two weeks after birth.

### 3.5. mRNA Levels Support mEGFP Expression Data

qPCR is used to verify the changes in expression pattern observed in the reporter mice at RNA level. The cornea, lens, and retina cannot be separated well at E11.5, so mRNA from wild-type eyes at other corresponding time points is analyzed, and E13.5 is used as the control. In general, PCR results are basically consistent with the obtained expression pattern data. PDGFR*α* mRNA levels in the cornea start low at E13.5 and E15.5, followed by a significant increase at E17.5 (Figure 5(a)). From birth to maturity, PDGFR*α* mRNA remains at a high level, confirming mEGFP expression patterns in the cornea. PDGFR*α* mRNA levels in the lens start high at embryonic time points and decrease significantly at P7, to fall gradually to a vestigial level at P60 (Figure 5(b)). However, mEGFP-positive cells decrease significantly at P14 in the lens. Nevertheless, qPCR remains high in agreement with mEGFP expression patterns. The qPCR data for the retina is also consistent with the mEGFP expression data. PDGFR*α* mRNA abundance starts at a very low level in early embryonic time points and increases gradually, reaching the peak at P1~P7 (Figure 5(c)). Once the eyelids start opening, PDGFR*α* mRNA levels decrease significantly and maintain such levels.

## 4. Discussion

Although several reports [19] have clarified the importance of PDGFR-A during the development of cornea, lens, and retina, the PDGFR*α*'s potential role has remained less clear in eye development. Our study provides PDGFR*α* expression maps with high spatial and temporal resolution and fate maps of PDGFR*α*-expressing cells. Moreover, we attempt to further explore the PDGFR*α*'s role in the progressive formation of the eye by blocking PDGFR*α* signals at postnatal stages.

While PDGFR*α* expression in the developing cornea has not been analyzed in detail before, and albeit, there are very few reports [19] on the PDGFR*α* expression during corneal development, the results herein provide new information about PDGFR*α* signaling in the cornea. In early studies [19] of in situ hybridizations, PDGFR*α* mRNA is found to be highly expressed in the corneal stroma and periocular mesenchyme (POM) in the E15 mouse eyes. The identity and fate of these cells, however, remain unknown. In our short-term tracing experiments, we observed that PDGFR*α* could be expressed in the cornea as early as E12.5, when the POM began to migrate into the space between the anterior epithelium of the lens vesicle (LV) and the surface ectoderm (SE). In our long-term tracing experiments, we, however, do not detect the PDGFR*α* expression in the corneal endothelial cells, although both the corneal endothelial and corneal stromal cells were derived from POM [18, 24].

From E11.5~E17.5, PDGFR*α*-expressing cells gradually increase to very high level and are highly expressed throughout the postnatal corneal development. Early reports, using PDGFR*α*-GFP mouse, found PDGFR*α* expression in the corneal stroma in adults [25]. However, in the current study, PDGFR*α* cells and their descendants are confined to the corneal stroma at all examined ages, and marker analyses uncover that these cells are keratocytes, the most abundant group of cells in the corneal stroma. In contrast to the mouse cornea, PDGFR*α* is found on the corneal stromal keratocytes, corneal endothelial cells, and, to a much lesser extent, on the epithelial cells in sections of human corneas [26]. Hence, attention should be payed to the different PDGFR*α* expression patterns among different species.

At embryonic and postnatal stages, we observed PDGFR*α*-expressing cells were localized to the lens epithelium and their differentiating lens fibers, partly in accordance with recent studies [19, 27]. However, a few differences might be pointed out. (1) Our short-term tracing experiments and immunostaining experiments indicated that PDGFR*α*-expressing cells were expressed at very early embryonic stages (E10.5), when the lens vesicle had just detached from the surface ectoderm and had a large central cavity. (2) PDGFR*α* expression had been restricted to the lens epithelium in our immunostaining experiments and previous studies using ISH or IHC [18, 27]. However, our long-term tracing experiments reveal that PDGFR*α*-expressing cells contribute to the lens epithelial and fiber cells. Therefore, in the differentiation process of the lens epithelial cells into fiber ones, the PDGFR*α* expression gradually decreases, or even stops. (3) As the lens continues to develop, the PDGFR*α*-expressing cells become more localized to the proliferating epithelial and fiber cells at the lens equator. Lens fiber cells in the posterior lens are not able to express PDGFR*α* in adults, even after long-term lineage tracing. The decline of PDGFR*α* expression in the fiber cells corresponds to the fiber cells' final differentiation process; the fiber cells lose their mitochondria and cell nuclei [3].

Our short-term tracing results concerning PDGFR*α* expression in the developing retina are in agreement with previous reports [20, 27], confirming the dynamic expression variation between different developmental stages. At early embryogenesis, PDGFR*α* is not expressed in the retina until E17.5. At E17.5~E18.5, PDGFR*α* expression is distributed in the centre of the retina. The mEGFP-positive cells in the centre of the retina's inner surface are astrocytes, instead of retinal ganglion cells (RGCs). These results conform to a previous report by Mudhar et al. [27], in which PDGFR*α* mRNA was observed at the optic nerve head (ONH) from E14 and spread across the retina's inner surface starting at E18. However, PDGFR*α* is not expressed in the retina until P1 in our immunostaining experiments. The difference between immunostaining experiments and short-term tracing experiments may be due to the fact that only a small number of cells in the nerve fiber layer expressed PDGFR*α* between E17.5 and E18.5, which are not detected by immunostaining. Interestingly, in our long-term tracing experiments, when eyes are harvested at P14 after a single dose of tamoxifen at E13.5 or E15.5, PDGFR*α* expression is detected in the retina's inner surface. Our results confirm the data by Mudhar et al. that the optic nerve head expresses PDGFR*α* from E14 and does not migrate to the retina at this time, whereas it will start to migrate around E18.

Postnatally, our findings on PDGFR*α* expression in the retina correspond with recent studies [27, 28]. PDGFR*α* expression in astrocytes in the nerve fiber layer persists throughout postnatal life into adulthood. Expression of PDGFR*α* significantly increases at P1~P7 and is associated with Sox9 and glutamine synthetase expression. A band of PDGFR*α*-expressing cells emerging in the INL is previously reported at P2. PDGFR*α*-expressing cells in the INL are most likely either bipolar neurons or Müller glia [27]. Our present data identifies a subpopulation of Müller glia cells in the INL, as cells expressing PDGFR*α* in the postnatal neural retina. No PDGFR*α* staining is visible in the INL of mice older than P14, which contradicts a previous study using PDGFR*α*-EGFP mice. Takahama et al. [25] reported that a subpopulation of amacrine cells in the inner nuclear layer expressed PDGFR*α* in the adult mouse retina. However, the number of these amacrine cells was very small, which may be the reason why we did not observe them.

Expectedly, PDGFR*α* mRNA levels do not fully match the expression of mEGFP. This is likely because mEGFP-positive cells represent PDGFR*α*-positive cells and their progeny cells, whereas these progeny cells may not express PDGFR*α*. Thus, mEGFP could be considered relevant as a contemporary or historic marker for PDGFR*α* expression. More studies are needed to comprehensively understand the PDGFR*α*'s expression pattern in the eye.

## 5. Conclusions

Our expression and lineage tracing studies with PDGFR*α* CreERT2; mT/mG mice provide a comprehensive map of the PDGFR*α* expression in various ocular lineages and identify the major cell types involved in PDGFR*α* signaling during eye development (Table 1). Our findings not only confirm the previously reported expression patterns but also add new information of cell fate.

## Figures and Tables

**Figure 1:** Cells expressing PDGFR*α* lineage in the adipose tissue, tail, kidney, liver, and adult eye (P60). Tamoxifen is administrated to an adult for 3 consecutive days and harvested at the seventh day. (a, e) Arrowheads point mEGFP staining in the adipose cells. (b, f) Arrowheads point mEGFP staining in the bone marrow stromal cells. (c, g) Arrowheads point mEGFP staining in the kidney mesangial cells. (d, h) Arrowheads point mEGFP staining in the hepatic stellate cells. (j–l) mEGFP-positive cells in the cornea, lens, and retina. (j) Arrowheads mark mEGFP-positive cells coexpressing ALDH3A1. (k) Arrows mark mEGFP-positive cells coexpressing *α*B-crystallin. (l) Hollow arrowheads mark mEGFP-positive cells coexpressing GFAP.

**Figure 2:** Cells expressing PDGFR*α* lineage in the embryonic eye. (a, e, i, and m) Tamoxifen is administrated at E11.5. (b, f, j, and n) Tamoxifen is administrated at E13.5. (c, g, k, and o) Tamoxifen is administrated at E15.5. (d, h, l, and p) Tamoxifen is administrated at E17.5. (a–h) Eyes are collected one day after tamoxifen administration. (i–p) Eyes are collected at P0. Arrowheads, arrows, and hollow arrowheads point mEGFP-positive cells in the cornea, lens, and retina, respectively.

**Figure 3:** Cells expressing PDGFR*α* lineage from the embryonic to the postnatal eye. (b–d) Eyes are administrated with tamoxifen at E11.5 and collected at P14. (f–h) Eyes are administrated with tamoxifen at E13.5 and collected at P14. (j–l) Eyes are administrated with tamoxifen at E15.5 and collected at P14. (n–p) Eyes are administrated with tamoxifen at E17.5 and collected at P14. Arrowheads, arrows, and hollow arrowheads mark mEGFP-positive cells coexpressing ALDH3A1, *α*B-crystallin, and GFAP, respectively.

**Figure 4:** Cells expressing PDGFR*α* lineage in the postnatal eye. (b–d) Eyes are administrated with tamoxifen at P1 and collected at P28. (f–h) Eyes are administrated with tamoxifen at P3 and collected at P28. (j–l) Eyes are administrated with tamoxifen at P7 and collected at P28. (n–p) Eyes are administrated with tamoxifen at P14 and collected at P28. (b, f, j, and n) mEGFP-positive cells are not coexpressing BRA3A (a ganglion cell marker). (c, g, k, and o) Hollow arrowheads mark mEGFP-positive cells coexpressing Sox9. (d, h, l, and p) Hollow arrowheads mark mEGFP-positive cells coexpressing glutamine synthetase.

**Figure 5:** PDGFR*α* gene expression. Cornea (a), lens (b), and retina (c) quantitative PCR results (mean + SEM) at different developmental time points. E13.5 is selected as a reference sample, and base values set at 1. Fold change is represented on the *y*-axis (2^−ΔΔCt^). ^∗^*P* < 0.05, two-way ANOVA, and Tukey's multiple comparisons test.

**Table 1:** Summary of the spatiotemporally specific contribution of the PDGFR*α*-expressing cells to the developing eye.

	Corneal stromal cells	Lens epithelial cells/fiber cells	Retinal astrocytes	Retinal Müller glial cells
E11.5	+	+++	-	
E13.5	+	+++	-	-
E15.5	++	+++	-	-
E17.5	+++	+++	+	-
P1	+++	+++	++	++
P3	+++	+++	+++	+++
P7	+++	+++	+++	+++
P14	+++	++	+++	-
P60	+++	+	+++	-

The (**+**) and (-) indicate the presence and absence of mEGFP-positive cells in the cornea, lens, and retina, respectively, with (**+++**) indicating highest levels of mEGFP-positive cells present.

## Data Availability

The datasets analyzed during the current study are available from the corresponding author on reasonable request.
